The article "Effect of Executive Dysfunction on Posture Control and Gait after Stroke" was published in 2021. Journal: Evid Based Complement Alternat Med.

# Effect of Executive Dysfunction on Posture Control and Gait after Stroke

**DOI:** 10.1155/2021/3051750

**Published:** 2021-10-12

**Authors:** Huixian Yu, Qianqian Zhang, Sihao Liu, Changbin Liu, Pei Dai, Yue Lan, Guangqing Xu, Hao Zhang

**Affiliations:** ^1^School of Rehabilitation, Capital Medical University, China Rehabilitation Research Center, Beijing 100068, China; ^2^Department of Rehabilitation Medicine, Beijing Tiantan Hospital, Capital Medical University, Beijing 100060, China; ^3^Department of Rehabilitation Medicine, Guangzhou First People's Hospital, School of Medicine, South China University of Technology, Guangzhou 510050, China; ^4^Department of Rehabilitation Medicine, Guangdong General Hospital, Guangdong Academy of Medical Sciences, Guangzhou 510080, China

## Abstract

**Objective:**

The purpose of the study was to observe the effects of executive dysfunction (ED) on gait and postural control during walking after stroke.

**Methods:**

In this study, 34 subjects with stroke and ED (8 women and 26 men; age, 55.41 ± 7.89 years; time since stroke onset, 1.3 ± 0.12 months) were recruited. Stroop color-word test (SCWT), 10-meter walk test (10MWT), timed-up-and-go test (TUGT), and gait analysis were evaluated. The correlation among the correct number of Stroop tasks (SCWT-C), the number of time-consuming tasks (SCWT-T), the amount of interference (SIE-M and SIE-T) and posture control, and gait-related parameters was analyzed.

**Results:**

The results indicated that SCWT-C was negatively correlated with 10MWT, TUGT, and bilateral symmetry (*P* < 0.05). However, there was no significant correlation between SCWT-C and stride (*P* > 0.05). A significant negative correlation was seen between SCWT-C and bilateral symmetry (*P* < 0.05). There was no significant correlation between SCWT-T and stride (*P* > 0.05). SCWT-T was positively correlated with TUGT, 10MWT, and bilateral symmetry (*P* < 0.05). SIE-T was positively correlated with TUGT and bilateral symmetry (*P* < 0.05). There was no significant correlation between SIE-T and 10MWT or stride (*P* > 0.05). SIE-M was positively correlated with TUGT and bilateral symmetry (*P* < 0.05). There was no significant correlation between SIE-T and 10MWT or stride (*P* > 0.05).

**Conclusions:**

ED is closely related to the decline in postural control and the occurrence of falls. In the early phases of stroke rehabilitation, physiotherapists should focus on the patients' executive function to accelerate the recovery of postural control.

## 1. Introduction

Hemiplegic gait is the most common sequela of stroke [1]. The difficulty in walking or shifting restricts the range of the patients' activities, increases the burden of the caregivers, and also affects the patients' psychology [2]. Functional community walking needs attention to aspects such as flexibility and multitasking [3]. The ability to switch between tasks or simultaneously perform multiple tasks is damaged after stroke. Therefore, falls may result from the inability to effectively allocate attention to posture control rather than balance dysfunction [4]. Attention and anti-interference are important components of executive function (EF). The prevalence of EF impairment was 49% amongst all stroke patients and 34% amongst those with excellent clinical recovery [5]. According to the existing statistics for patients in the early stage (<3 months) of stroke, the incidence rate of executive dysfunction (ED) is quite high. ED is a common poststroke cognitive symptom and compromises the patients' independence in daily activities. Previous studies have often relied on brief cognitive tests without fully considering the wide spectrum of EF subdomains [6]. After stroke, people with ED may show worse balance due to difficulty performing novel, targeted activities, such as standing up and moving from bed to chair [7]. In China, most cognitive rehabilitation and physical rehabilitation in rehabilitation facilities are separate. Physiotherapists seldom pay attention to the influence of patients' cognitive components on balance function during physical rehabilitation.

Hence, this study aimed to recruit poststroke patients with ED, conduct gait analysis, walk test, and timed-up-and-go test, and analyze the correlation of ED with gait parameters and stand up and walk test. Furthermore, this research intended to observe the effects of ED on gait and postural control during walking after stroke.

## 2. Methods

### 2.1. Participants

We collected the data of 34 patients (8 women and 26 men; age, 55.41 ± 7.89 years; time since stroke onset, 1.3 ± 0.12 months) with hemiplegic gait developed after stroke and who had visited the department of rehabilitation medicine, Beijing Tiantan Hospital, Capital Medical University, from November 2020 until June 2021. The patient inclusion criteria were as follows: (1) the definitive diagnosis of the first-ever stroke; (2) right or left basal ganglia region stroke; (3) age of 40–60 years, either male or female sex; (4) ≤3 months poststroke; (5) >12 years of education; (6) MoCA score of 20–30; (7) lower-limb Fugl–Meyer motor assessment score of 20–30; and (8) the ability to walk for 10 m without help. The exclusion criteria were as follows: (1) other cerebrovascular diseases; (2) sensory aphasia; (3) traumatic hemorrhage; (4) sensory impairment; (5) combination with other osteoarticular system diseases; and (6) failure to cooperate with the inspection process.

The Ethics Committee of Beijing Tiantan Hospital Affiliated to the Capital Medical University approved this study. All participants provided their written informed consent before data collection. The study was conducted in accordance with the Declaration of Helsinki.

### 2.2. Screening Measures

1. Montreal Cognitive Assessment (MoCA): MoCA is a rapid screening assessment tool used for cognitive dysfunction. It included 11 items from across eight cognitive areas, including attention and concentration, executive function, memory, language, visual structure skills, abstract thinking, computation, and orientation. Patients with scores ranging from 20 to 30 points were recruited.
2. 10 m walking test (10MWT): for this test, the patients were required to walk along a corridor of >10 m, with two invisible marking lines made at either end of the distance of the walking path. The time to test began with the first step of the marking line and ended when the second marking line was crossed.
3. Timed-up-and-go test (TUGT): for the TUGT, during the evaluation, the patients were asked to remain seated in an armrest chair (seat height 45 cm, armrest height 20 cm), with the body leaning against the back of the chair and hands resting on the armrest. Next, a cone was placed on the floor 3 m away from the seat. When the experimenter gave the “go” command, the patient was required to stand up from the armchair. After standing firmly, the patient would walk for 3 m forward with the usual walking gait, turn around the cone, walk back to the chair, and then turn to sit down and lean back. No physical assistance was allowed during the test [8].
4. Plantar pressure center of pressure (COP) of the gait analysis test: the patient was allowed to walk naturally on the plantar pressure plate and maintain the stride. The distance difference between the left-right swing of the center of gravity transfer trajectory (bilateral symmetry of COP) was recorded. The normal pressure trajectory of the center of gravity is a “butterfly” distribution, with the left-right symmetry, and the difference in the left-right swing amplitude was 0. The “butterfly” type of hemiplegic gait becomes atypical or even disappears (as shown in Figure 1).
5. The Stroop color-word test (SCWT): it was divided into the following three steps: (i) in the first step, card A was presented, which consisted of four types of color words (i.e., yellow, red, blue, and green). A total of 50 words were read out as quickly and correctly as possible. (ii) Next, card B was presented, which consisted of dots in four different colors (i.e., yellow, red, blue, and green). (iii) Finally, card C was presented, and the above four-color words were printed in four different colors. The subjects were asked to try to read out the color of the words as quickly and correctly as possible, rather than thinking about the meaning of the words. The analysis indicators included the amount of time taken to complete reading each card, the number of correct readings, and the number of mistakes, among others. Stroop interference effects (SIE) indicators are as follows:
6. SIE time (SIE-T) = time of card C − time of card B;
7. SIE mistake count (SIE-M) = mistake number of card C − mistake number of card B.

The larger the SIE, the lower was the interference inhibition efficiency.

### 2.3. Data Analysis

Statistical analysis and graphing were performed using GraphPad Prism 8.0 (GraphPad Software, Inc., San Diego, California, USA). Continuous variables were expressed as mean ± standard deviation. Correlations between SCWT time (SCWT-T), SCWT correct count (SCWT-C), SIE-T, SIE-M, and the posture change, as well as the gait, were analyzed by Pearson bivariate correlation analysis. *P* < 0.05 was considered to be statistically significant.

## 3. Results

The participant characteristics are presented in Table 1. The mean time since stroke onset was 1.3 ± 0.12 months (range, 0–3 months). The mean score of MoCA was 25.78 ± 8.19 (range, 20–30). The mean lower-limb Fugl–Meyer motor assessment score was 24.56 ± 10.54(range, 20–28).

Correlation of SCWT-C with 10MWT, TUGT, stride, and bilateral symmetry of COP (Figure 2): the result showed significant negative correlation between SCWT-C and 10MWT (*R*^2^ = 0.666, *P* = 0.001) and moderately negative correlation between SCWT-C and TUGT (*R*^2^ = 0.383, *P* ≤ 0.001). There was no significant correlation between SCWT-C and stride (*R*^2^ = 0.045, *P* = 0.230). A moderately negative correlation was present between SCWT-C and bilateral symmetry (*R*^2^ = 0.353, *P* = 0.002).

Correlation of SCWT-T with 10MWT, TUGT, stride, and bilateral symmetry of COP (Figure 3): there was no significant correlation between SCWT-T and 10MWT (*R*^2^ = 0.001, *P* = 0.900). However, a moderately positive correlation was seen between SCWT-T and TUGT (*R*^2^ = 0.289, *P* = 0.001). There was no significant correlation between SCWT-T and stride (*R*^2^ = 0.008, *P* = 0.613). Furthermore, a moderately positive correlation was observed between SCWT-T and bilateral symmetry (*R*^2^ = 0.249, *P* = 0.003).

Correlation of SIE-T with 10MWT, TUGT, stride, and bilateral symmetry of COP (Figure 4): there was no significant correlation between SIE-T and 10MWT (*R*^2^ = 0.001, *P* = 0.938). The result suggested a moderately positive correlation between SIE-T and TUGT (*R*^2^ = 0.355, *P* = 0.002). There was no significant correlation between SIE-T and stride (*R*^2^ = 0.038, *P* = 0.269). A moderately positive correlation was noted between SIE-T and bilateral symmetry (*R*^2^ = 0.389, *P* ≤ 0.001).

Correlation of SIE-M with 10MWT, TUGT, stride, and bilateral symmetry of COP (Figure 5): there was no significant correlation between SIE-M and 10MWT (*R*^2^ = 0.011, *P* = 0.558). The findings implied a moderately positive correlation between SIE-M and TUGT (*R*^2^ = 0.387, *P* ≤ 0.001). There was no significant correlation between SIE-M and stride (*R*^2^ = 0.042, *P* = 0.244). Nonetheless, a significant positive correlation was seen between SIE-M and bilateral symmetry (*R*^2^ = 0.520, *P* ≤ 0.001).

## 4. Discussion

ED seriously affects the quality of life of the patients [9–11]. It is the core and first symptom of cognitive impairment [12], and its impact is comparable to that of limb dysfunction as it hinders the comprehensive rehabilitation of the patients [9]. ED also affects the activities of daily living (ADL), social participation, work performance, functional prognosis, and return to work [13]. Compared with normal patients, people with ED may show worse balance due to difficulty performing novel, targeted activities, such as standing up and moving from bed to chair. EF is a group of higher cognitive functions that control or monitor other low-level functions to achieve a selected goal. These functions include working memory, inhibitory control, attentional control, cognitive flexibility, reasoning, planning, concept formation, and problem-solving [14, 15]. It is generally agreed that there are three core EFs, namely, inhibitory control (including behavioral inhibition executive dysfunction) and interference control (selective attention and cognitive inhibition), working memory (WM), and cognitive flexibility.

ED is the reduced ability to do something, and the decline or loss of problem-solving ability is the main feature. ED can be divided into the following three aspects: initiation, termination, and self-regulation disorder [16]. The brain areas related to EF include the prefrontal-striatal circuit and the cerebellum, among which the prefrontal-striatal circuit also includes the dorsolateral prefrontal lobe, orbitofrontal lobe, anterior cingulate gyrus, and basal ganglia [17]. Patients with stroke who have infarction or hemorrhage in the above locations tend to exhibit significant ED.

Our present understanding of cognitive-motor networks and the influence of cognition on movement, gait characteristics, and postural control is limited. The existing research findings on the effect of cognition on gait speed and stride are controversial [18, 19]. The present study demonstrated a significant positive correlation between SCWT-T and 10MWT. Nevertheless, we did not see significant correlations between 10MWT and SCWT-C or SIE. The correlation analysis among SCWT, SIE, and stride length did not show any significance. In the process of walking in a straight line, muscle strength, endurance, and coordination may be more important than attention and posture control.

Falls after stroke are common [20]. Many studies have established a high correlation between TUGT and fall-risk prediction [21]. In this study, there were significant correlations between TUGT and SCWT (SCWT-T, SCWT-C, SIE-T, and SIE-M). Unlike walking along a straight line, in the TUGT, the complex control of the center of the body weight in getting up, walking, stopping, turning around, and sitting down requires more cognitive resources. In the analysis of central pressure, we found that the curve of people with cognitive dysfunction was more asymmetric and that the force line was more disordered. Instead of the normal straight-line distribution, the central pressure was curved, which meant that these patients had a poorer center of gravity control, higher energy consumption during walking, and a more unsteady gait. This study revealed the strong correlation between EF and the distribution of COP. Gait variability and symmetry are commonly used as quantifiable measures of mobility. COP trajectory during walking is commonly represented using the butterfly diagram. Previous research used the butterfly diagram to present essential gait characteristics, such as variability, stride width, and symmetry between legs [22]. Asymmetrical gait features are more significant. SCWT is a test developed by Stroop in 1935 to study the influence of interference. This test is often employed in the evaluation of EF in scientific research and clinical practice and is of great significance in the early detection of EF impairment. SCWT is a test of attention, and SIE reflects the dominant inhibitory component of EF. This research signified that decreased inhibition and attentional ability could reduce postural control and center of gravity control. Asymmetrical gait features are more significant.

In this study, there was no significant correlation between SCWT and step length or speed. Executive function is more affected by postural shift, while straight walking may require fewer cognitive resources.

In the past decade, conventional stroke rehabilitation has encompassed a spectrum of evidence-based exercise training interventions that involve improving strength, flexibility, endurance, balance, and gait [23]. Previously, studies have exploited repetitious and intense balance training to improve clinically relevant fall-risk predictors and balance confidence. However, systematic reviews (SRs) and meta-analyses have found that virtual reality-based training is more effective in improving clinical balance measures [24]. After the stroke, the patients' ability to perform other tasks during walking is lowered or even lost completely, and the ability to notice obstacles and avoid them is decreased, which results in falls.

Many factors lead to falls in stroke patients, and the major ones are abnormal walking patterns, impaired balance function, and poor postural control. Postural control requires multiple sensory inputs, which are processed by the central nervous system and executed by the motor system. A framework for the study of postural control has been proposed, which includes biomechanical factors, spatial orientation, motor strategy, dynamic control ability, sensory strategy, and cognitive processing [25]. An SR on the effects of balance and motor function rehabilitation (248 primary studies and 10,638 participants) showed a defective result. A wide variety of balance and postural control outcomes were included. It was observed that 61% of the SRs focused on the effectiveness of physical therapy, 20% on virtual reality, 6% on electromechanical devices, 4% on Tai-Chi, whole-body vibration, and circuit training intervention, and 2% on cognitive rehabilitation [26]. The findings suggested that cognition is not sufficiently valued in balance function and motor rehabilitation. Recently, mounting evidence has indicated that cognitive function is involved in complex motor and posture control and that posture control during walking receives instructions from the cognitive regions of the brain [27]. The basal ganglia are a common stroke site and an important part of the execution-motor functional brain network [28]. This study identified that the incidence of early EF impairment after basal ganglia stroke is very high and that it tends to affect the patients' posture control ability, thereby increasing the occurrence of falls.

## 5. Conclusions

Our study demonstrated the strong correlation between EF and postural control in early of stroke. Furthermore, the findings suggested that impaired early ED is associated with a high fall rate in the early stage of stroke. In the early phases of stroke rehabilitation, physiotherapists should focus on the patients' ED to accelerate the recovery of postural control. In the next study, we aspire to perform early EF intervention for patients with stroke and observe the improvement in posture control ability. We hope to conduct more in-depth research on brain imaging and brain network analysis.

## Figures and Tables

**Figure 1:** (a) The normal central pressure trajectory is of butterfly distribution, with a left and right cross symmetry and each gait cycle almost overlapping straight lines. (b) The pressure lines of stroke patients were asymmetric, and the closer to the affected side, the more disordered they were, and the pressure lines of each gait cycle did not overlap.

**Figure 2:** Correlation of SCWT-C with 10MWT, TUGT, stride, and bilateral symmetry of COP; SCWT-C and 10MWT, a significant negative correlation; SCWT-C and TUGT, a significant negative correlation; SCWT-C and stride, no significant correlation; SCWT-C and bilateral symmetry, a significant negative correlation.

**Figure 3:** Correlation of SCWT-T with 10MWT, TUGT, stride, and bilateral symmetry of COP; SCWT-T and 10MWT, no significant correlation; SCWT-T and TUGT, a significant positive correlation; SCWT-T and stride, no significant correlation; SCWT-T and bilateral symmetry, a significant positive correlation.

**Figure 4:** Correlation of SIE-T with 10MWT, TUGT, stride, and bilateral symmetry of COP; SIE-T and 10MWT, no significant correlation; SIE-T and TUGT, a significant positive correlation; SIE-T and stride, no significant correlation; SIE-T and bilateral symmetry, a significant positive correlation.

**Figure 5:** Correlation of SIE-M with 10MWT, TUGT, stride, and bilateral symmetry of COP; SIE-M and 10MWT, no significant correlation; SIE-M and TUGT, a significant positive correlation; SIE-M and stride, no significant correlation; SIE-M and bilateral symmetry, a significant positive correlation.

**Table 1:** Demographic characteristics of the participants.

Age (years)	Hemiplegic limb (number)		Onset time (M)	Sex (n)		Type of stroke		Fugl–Meyer	MoCA
	Left	Right		F	M	Inf.	Hem.		
55.41 ± 7.89	19	15	1.3 ± 0.12	8	26	24	10	24.56 ± 10.54	25.78 ± 8.19

## Data Availability

The data used in this study can be obtained by contacting the corresponding author.
